# Pain control for patients with hepatocellular carcinoma undergoing CT-guided percutaneous microwave ablation

**DOI:** 10.1186/s40644-018-0174-4

**Published:** 2018-11-01

**Authors:** Hong-Zhi Zhang, Jie Pan, Jing Sun, Yu-Mei Li, Kang Zhou, Yang Li, Jin Cheng, Ying Wang, Dong-Lei Shi, Shao-Hui Chen

**Affiliations:** 1 Department of Radiology, Peking Union Medical College Hospital, Peking Union Medical College, Chinese Academy of Medical Sciences, No. 1 Shuaifuyuan, Dongcheng District, Beijing, 100730 China; 2 Department of Anesthesiology, Peking Union Medical College Hospital, Peking Union Medical College, Chinese Academy of Medical Sciences, Beijing, China

**Keywords:** Microwave ablation, Hepatocellular carcinoma, Pain, Analgesia, Morphine

## Abstract

**Background:**

Hepatic percutaneous microwave ablation (MWA) is usually performed in patients under conscious sedation. Nonetheless, many patients reported pain during the procedure. The current study investigated the safety and effectiveness of analgesia given at personalized dosage during the MWA procedure.

**Methods:**

A total of 100 patients with hepatocellular carcinomas (HCCs) were included in this study. These patients underwent CT-guided percutaneous MWA between February and October 2017. Patients were randomized into two groups: Experimental group (*n* = 50) and Control group (n = 50). Patients in the Control group were given 5 mg of morphine intravenously, followed by 10 mg of morphine injected subcutaneously 30 min before surgery. Patients in the Experimental group were given a personalized dosage of morphine during the procedure when the Visual Analogue Scale (VAS) was ≥4. Other clinical and treatment parameters were also analysed.

**Results:**

A significantly less amount of morphine (*p* < 0.001) was used in the experimental group (7.18 ± 1.65 mg) than in the control group (17.40 ± 2.52 mg). No significant differences were found in the number of patients who needed to discontinue the surgery (*p* = 0.242). Other clinical parameters including heart rate, systolic and diastolic blood pressures at various time points were comparable. Importantly, a lower VAS was reported in the experimental group, indicating a lower pain intensity experienced by patients during the procedure.

**Conclusion:**

The administration of personalized dosage of morphine to HCC patients undergoing percutaneous MWA is an effective and safe procedure for pain control.

## Introduction

Tumor ablation is defined as the direct application of chemical or thermal therapies to tumor to achieve substantial tumor destruction or eradication; and microwave ablation (MWA) has been recognized as an alternative treatment for patients with hepatocellular carcinoma (HCC). MWA may be used when the curative treatments of HCC (e.g. surgical resection or liver transplant) could not be performed. Studies reported that only 10–54% of all HCC patients were eligible for the curative surgical treatments [1–3]. Other clinical parameters including heart rate, and the difficulties with the surgical resection were related to the site, size, number of tumors, as well as the extrahepatic involvement and remaining liver function [4, 5]. MWA has become another choice to the treatment of HCC, providing effective and reproducible local tumor control and minimal morbidity [6, 7]. Additionally, MWA was a relatively low-risk and minimally invasive procedure for liver tumors [6, 7].

A conscious sedation and local anesthesia were usually sufficient for percutaneous CT-guided MWA, since the operation time of the MWA treatment was short, about 5 to 15 min [8]. However, many patients reported pain during and/or after the treatment [9, 10]. The risk of having at least moderate pain after the treatment may be related to the ablation volume and time and post ablation increase in AST level [9]. The visceral pain caused by the thermal effects of the microwave could be severe, resulting in an uneven respiratory rate and increased surgical risk. For patients who are expected to have a long MWA procedure (e.g. 3 h or longer), a general anesthesia may be preferred.

As variations were seen in perceived pain and discomfort during the procedure, it is important to personalize the pain control strategy. An effective pain control strategy would allow a smooth operation. Conscious analgesic sedations, such as fentanyl, droperidol, midazolam, were used in a standard dose across patients [8, 11]. The current study investigated the outcome of pain control between patients using a standard versus personalized dose of morphine under local anesthesia. We also provided recommendations for the pain control strategy in HCC patients receiving MWA procedure.

## Patients and methods

### Patients

A total of 100 HCC patients receiving CT-guided MWA treatment between February and October 2017 were included in this study. All patients had a single lesion of HCC < 3 cm, and a single probe was used for the ablation. All patients had no cognitive and speech impairment, and no hearing or cerebrovascular diseases. The MWA was performed at 50–70 W for 5–6 min. The insertion of water-cooled microwave ablation needles (Nanjing Vision-China Medical Devices R&D Center, China) was performed under the guidance of real-time CT scans.

Medical information, including body weight, long-term drinking history, long-term use of analgesic drug history, history of allergies, hypertension and coronary heart disease were recorded. The number and diameter of HCC tumors were also recorded. This study has been approved by our institute’s Ethics committees. All patients provided written informed consent.

### Methods of analgesia

Patients were randomized into two groups: Experimental group (*n* = 50) and Control group (*n* = 50). The pain intensity was assessed for all patients before and during surgery using Visual Analogue Scale (VAS), ranging from ‘0’ representing no pain to ‘10’ representing worst pain imaginable [12]. Patients were given 8 mg intravenous injection of ondansetron hydrochloride and 5 mg of dexamethasone (Northeast Pharmaceutical Group Shenyang No. 1 Pharmaceutical. Co. Ltd., China) 30 min before surgery to prevent and alleviate nausea. During the surgery, injection of morphine or 2% lidocaine for skin puncture were used for anaesthesia.

Patients in the Control group were given 5 mg of morphine intravenously, followed by 10 mg of morphine injected subcutaneously 30 min before surgery. For patients in the Experimental group, the first dose of morphine was given at a dose calculated from the body weight at 0.1 mg/kg and was given subcutaneously during the procedure when the VAS was ≥4. If additional morphine was needed during the procedure, a fixed dose at 5 mg was given in both groups. Naloxone hydrochloride (0.4 mg) and simple respirator were prepared and given to patients only when needed. Patients were accompanied by a nurse during the procedure.

### Evaluation

Vital signs including blood pressure, pulse rate, heart rate, and respiration rate were recorded before and after surgery. Oxygen saturation and the mental status were also recorded. During the surgery, the presence of nausea and vomiting and the number of times and doses of morphine used, were recorded. VAS evaluation was performed in post-initiation of ablation at 0.5 min, 1.5 min, 2.5 min, 3.5 min, 4.5 min, 5.5 min.

### Statistical analyses

The SAS 9.3 was used for statistical analysis. Two-tailed test was used and *p* < 0.05 was considered as statistically significant. Categorical variables were presented in frequency (%); Chi-square test and Fisher’s exact test were used for comparisons between groups. Continuous variables were presented as mean ± standard deviation; Student’s t-test was used for analysis when the data were in normal distribution, or Wilcoxon rank-sum test was used. Two-way repeated measures ANOVA was used to compare intraoperative vital signs and pain score between two groups, and one-way repeated measures ANOVA was used for comparison within the group. The pre-operative vital signs and the pain score at 0.5 min of the ablation were used as baseline for comparison.

## Results

The baseline clinical characteristics, including sex, age, weight, comorbidity, size and anatomical location of the lesions, were summarized in Table 1. There were no significant differences in these parameters between the control and experimental groups.

**Table 1:** Comparison of baseline clinical characteristics between the two groups

Characteristics	Control Group	Experimental Group	*p*-value
	*n* = 50	*n* = 50	
Gender, n (%)			0.822
Male	13 (26.00)	14 (28.00)	
Female	37 (74.00)	36 (72.00)	
Hypertension, n (%)			0.106
Absent	41 (82.00)	34 (68.00)	
Present	9 (18.00)	16 (32.00)	
Coronary heart disease, n (%)			0.059
Absent	49 (98.00)	43 (86.00)	
Present	1 (2.00)	7 (14.00)	
Age (year), mean ± SD	60.3 ± 10.5	60.18 ± 11.71	0.896
Weight (kg), mean ± SD	68.48 ± 5.89	66.64 ± 10.57	0.286
Diameter of the largest lesion (cm)^a^, mean ± SD	2.14 ± 0.96	2.08 ± 0.96	0.275
Distance between the lesion and liver surface (cm)^a^, mean ± SD	2.78 ± 0.96	2.96 ± 1.16	0.343
Distance between the lesion and central hilar (cm)^a^, mean ± SD	3.87 ± 1.23	4.07 ± 1.33	0.462

^a^Two missing cases in the control group (*n* = 48)

The ablation treatment parameters and morphine usage were compared between the two groups (Table 2). The average time used for the ablation procedure was similar between the groups (control group: 5.33 ± 0.62 min vs. experimental group: 5.41 ± 1.04 min, *p* = 0.751). Various outputs (50 W, 60 W, 70 W) were used for the ablation. All of the patients in the control groups used the 50 W probe, while most of the patients in the experimental group used the 50 W or 60 W probes, with one patient used the 70 W probes (*p* < 0.001). In the experimental group, morphine was injected at various time points when VAS was ≥4 (6 patients at 0.5 min; 21 patients at 1.5 min; 12 patients at 2.5 min; 6 patients at 3.5 min); an average of 6.48 ± 1.01 mg of morphine was used for the first injection. Five patients (out of 50) had no morphine injection during the whole procedure (as the VAS was < 4). In the control group, 24 patients needed additional morphine injection during the procedure, while only 3 patients in the experimental group needed additional injection (*p* < 0.001). Overall, a significantly less amount of morphine (*p* < 0.001) was used in the experimental group (7.18 ± 1.65 mg) than in the control group (17.40 ± 2.52 mg). No significant differences were found in the number of patients who needed to discontinue the surgery (*p* = 0.242).

**Table 2:** Comparison of treatment parameters and morphine usage between groups

Treatment parameters and Morphine usage	Control Group	Experimental Group	*p*-value
	n = 50	*n* = 50	
Ablation duration, mean ± SD	5.33 ± 0.62	5.41 ± 1.04	0.751
Ablation probes			< 0.001
50 W	50 (100.00)	28 (56.00)	
60 W	0 (0.00)	21 (42.00)	
70 W	0 (0.00)	1 (2.00)	
Dose level of morphine in the first administration, experimental group, (mg), mean ± SD	–	6.84 ± 1.01^a^	–
Number of patients needed additional morphine during surgery	24(48.00)	3 (6.67)	< 0.001
Total amount of morphine used (mg)	17.40 ± 2.52	7.18 ± 1.65^a^	< 0.001
Number of patients with surgery terminated	3 (6.00)	0 (0.00)	0.242

^a^Morphine was given to 45 patients in the Experimental group who reported VAS ≥ 4, and 5 patients had no morphine administrated during the whole procedure

We used VAS as a tool to assess the pain intensity of patients during the procedure (Table 3). Overall, both of the groups had a significantly lower VAS at various time points (1.5 min, 2.5 min, 3.5 min, 4.5 min, 5.5 min post-initiation of ablation) when compared to the baseline within the group at 0.5 min post-initiation of ablation (*p* < 0.001). When compared across the groups, a significantly lower VAS was found in the experimental group at various time points (0.5 min, 1.5 min, 2.5 min, 3.5 min, 4.5 min, 5.5 min post-initiation of ablation), indicating patients experienced a lower pain intensity during the whole treatment procedure.

**Table 3:** VAS evaluation of the two group of patients at various time points of the ablation

Time points Post initiation of ablation	Control Group	Experimental Group	*p*-value ^a^
	*n* = 50	*n* = 50	
0.5 min	2.04 ± 1.97	1.02 ± 1.45	0.004
1.5 min	3.98 ± 1.95^c^	3.06 ± 1.27^b^	0.006
2.5 min	4.86 ± 1.7^c^	3.48 ± 1.30^b^	< 0.001
3.5 min	5.18 ± 1.62^c^	3.16 ± 1.20^b^	< 0.001
4.5 min	4.94 ± 1.64^c^	2.60 ± 1.09^b^	< 0.001
5.5 min	4.70 ± 1.46^c^	2.24 ± 0.85^b^	< 0.001
5 min after surgery	0.16 ± 0.55^c^	0.02 ± 0.14^b^	0.083
*p*-value	<0.001	<0.001	–

^a^Comparison between groups; ^b^Comparison within groups; ^c^Compared to 0.5 min of the Experimental Group and the *p*-values were < 0.05

Other clinical parameters including heart rate, systolic and diastolic blood pressures at various time points were also compared between the two groups, and no significant differences were found (Table 4, 5 and 6).

**Table 4:** Heart rate (mean ± SD, beats/ min) of the two groups of patients at various time points of the surgery

Time points Post initiation of ablation	Control Group	Experimental Group	*p*-value ^a^
Before Surgery	70.56 ± 8.18	72.52 ± 10.37	0.437
Before initiation of ablation	71.84 ± 8.98^c^	74.06 ± 10.96^b^	0.271
0.5 min	72.88 ± 7.84^c^	74.64 ± 11.87^b^	0.384
1.5 min	74.58 ± 9.91^c^	74.48 ± 12.61	0.965
2.5 min	75.32 ± 10.57^c^	74.42 ± 12.3	0.696
3.5 min	76.52 ± 11.15^c^	73.37 ± 11.87	0.176
	77.33 ± 12.02^c^	73.79 ± 10.96	0.135
5.5 min	78.89 ± 12.29^c^	73.98 ± 9.69	0.044
5 min after surgery	73.22 ± 7.77^c^	71.86 ± 9.53	0.436
*p*-value	< 0.001	0.046	–

^a^Comparison between groups; ^b^Comparison within groups; ^c^Compared to Experimental Group before surgery, and the *p*-values were < 0.05

**Table 5:** Systolic blood pressures (mean ± SD, mmHg) of the two groups of patients at various time points of the surgery

Time points Post initiation of ablation	Control Group	Experimental Group	*p*-value ^a^
Before Surgery	132.44 ± 11.83	135.22 ± 16.91	0.343
Before initiation of ablation	135.88 ± 12.41^c^	137.48 ± 18.27^d^	0.610
0.5 min	140.22 ± 13.58^c^	138.84 ± 20.07	0.688
1.5 min	142.94 ± 14.72^c^	142.4 ± 20.39^d^	0.880
2.5 min	144.36 ± 17.91^c^	143.84 ± 20.61^d^	0.893
3.5 min	146.02 ± 18.13^c^	145.16 ± 19.68^d^	0.822
4.5 min	146.06 ± 18.4^c^	144.63 ± 19.05^d^	0.708
5.5 min	147.05 ± 18.31^c^	142.21 ± 19.12^d^	0.235
5 min after surgery	136.50 ± 12.52^c^	138.34 ± 17.58	0.548
*p*-value	< 0.001	< 0.001	–

^a^Comparison between groups; ^b^Comparison within groups; ^c^Compared to Control Group before surgery, and the *p*-values were < 0.05. ^d^Compared to Experimental Group before surgery, and the *p*-values were < 0.05

**Table 6:** Diastolic blood pressures (mean ± SD, mmHg) of the two groups of patients at various time points of the surgery

Time points Post initiation of ablation	Control Group	Experimental Group	*p*-value ^a^
Before Surgery	74.40 ± 8.65	72.50 ± 8.95	0.283
Before initiation of ablation	76.98 ± 8.22^c^	74.10 ± 10.74^d^	0.610
0.5 min	79.30 ± 9.25^c^	75.9 ± 9.76^d^	0.688
1.5 min	79.08 ± 10.20^c^	78.52 ± 10.46^d^	0.880
2.5 min	81.62 ± 11.83^c^	78.42 ± 9.94^d^	0.893
3.5 min	80.98 ± 12.03^c^	77.14 ± 9.39^d^	0.822
	82.15 ± 11.04^c^	78.27 ± 9.28^d^	0.708
5.5 min	82.11 ± 11.16^c^	76.00 ± 8.32^d^	0.235
5 min after surgery	76.74 ± 7.99	73.96 ± 7.92	0.548
*p*-value	< 0.001	< 0.001	–

^a^Comparison between groups; ^b^Comparison within groups; ^c^Compared to Control Group before surgery, and the p-values were < 0.05. ^d^Compared to Experimental Group before surgery, and the *p*-values were < 0.05

## Discussion

Pain experienced during the ablation procedure is categorized in the side effect category, according to the guidelines for the standardization of terminology and reporting criteria for image-guided tumor ablation [13]. The intraoperative pain may affect the completion of a standardized treatment protocol. It has been reported that pain may be related to the side of the lesion and the amount of tissue necrosis [14], but the level of pain was unpredictable.

We found the administration of personalized dosage of morphine during the percutaneous CT-guided MWA treatment was an effective and safe procedure for pain control in HCC patients undergoing local anaesthesia. Local anaesthesia is commonly used for the tumor ablation procedure, since the operation time is usually short [8]. General anaesthesia may be indicated for patients with a low tolerance for pain, or patients with a history of alcohol or drug abuse. However, the general anaesthesia would require a more extensive preoperative evaluation of patients, special technicians (e.g. anaesthetists) and equipment. Importantly, there is a higher risk for patients undergoing general anaesthesia. The pain control strategy discussed in this study may provide a way to expand the patient population that could receive CT-guided MWA under conscious sedation.

Our study found that patients in the experimental group received a significantly less amount of morphine when compared to the control group. Patients with thermal ablation of subcapsular or hilar lesions may require higher doses of analgesics [15]. In our study, patients’ lesion locations with respect to central hilar and to the liver surface were comparable between groups, further suggesting the personalized dosage of morphine was at least equally effective. The reduced use of morphine could help to reduce the side effects (e.g. nausea, vomiting, blood pressure, respiratory depression, etc.) [16]. In addition, this pain control strategy was safe. The vital signs and cases of surgery termination were comparable between the two groups.

The analgesic method used in the experimental group provided a satisfactory pain control. Conventionally, morphine was given before the insertion of needles [17]; depending on the tumor location, size, the position of the needle inserted, repeated scanning and adjustment of the needle angle may be needed, resulting further pain. Therefore, it is important to have a prompt administration of analgesia through a timely evaluation of pain during the procedure. In addition to the VAS, other pain related parameters could be considered for assessing pain, such as the pain-related behaviours (facial expressions and postures), physiologic indicators (heart rate, blood pressure, respiratory rate).

The non-pharmacological methods of pain control, such as distraction, simple massage, and family support also helped to relive pain. A study reported that the non-pharmacological interventions used by ICU nurses complementary to pharmacological treatment could maximize the pain relief [18]. In our study, we also found that the support from nurses was important; it sometime helped to decrease the pain level perceived by patients.

## Conclusion

We showed that the administration of personalized dosage of morphine to HCC patients undergoing percutaneous MWA is an effective and safe procedure for pain control.

## Abbreviations

HCC: hepatocellular carcinoma
MWA: microwave ablation
VAS: Visual Analogue Scale
